The article "Impact of Zinc to Copper Ratio and Lipocalin 2 in Obese Patients Undergoing Sleeve Gastrectomy" was published in 2022. Journal: Biomed Res Int.

# Impact of Zinc to Copper Ratio and Lipocalin 2 in Obese Patients Undergoing Sleeve Gastrectomy

**DOI:** 10.1155/2022/9278531

**Published:** 2022-06-10

**Authors:** Hala M. Demerdash, Ahmed A. Sabry, Omar E. Arida

**Affiliations:** ^1^Department of Clinical Pathology, Alexandria University Hospitals, Alexandria University, Alexandria, Egypt; ^2^Department of Surgery, Faculty of Medicine, Alexandria University, Alexandria, Egypt; ^3^Department of Anaesthesia and Intensive Care, Medical Research Institute, Alexandria University, Alexandria, Egypt

## Abstract

Worldwide, obesity constitutes a significant health issue. There is the perception that obesity is influenced by subclinical inflammation caused by trace elements (TE). Lipocalin 2 (Lcn2) is an adipokine that is abundantly expressed in adipose tissue, largely in response to metabolic stress; TE deficiency is expressed in metabolic dysfunction as increased oxidative stress, the development of dyslipidaemia and insulin resistance. The primary aim of this study is to explore the relationship between Lcn2 inflammatory biomarkers and the TE status of subjects with morbid obesity who are undergoing laparoscopic sleeve gastrectomy (LSG); the secondary aim is to evaluate the Zn-to-Cu ratio in those with a detected TE deficiency. When this prospective cohort study was conducted, 107 subjects with morbid obesity (i.e., 69 women, 38 men) ranging in age from 20 to 55 years were recruited. Anthropometric measurements and laboratory investigations were performed preoperatively and nine months postoperatively; and blood samples were collected to determine the subjects' iron, Zn, Cu, Lcn2, and other inflammatory biomarkers. The results revealed 16.82% of the subjects exhibited preoperative Zn deficiency, which increased to 22.43% postoperatively; none of studied subjects exhibited Cu deficiency in the two consecutive measurements; and the 10.28% preoperative prevalence of iron deficiency increased to 15.89% postoperatively. While a negative correlation was observed between the delta body weight change and Lcn2, leptin, and HOMA-IR, a positive correlation was observed between the delta body weight change and the Zn-to-Cu ratio. These findings suggest the existence of preoperative obesity is associated with inflammatory status that may be triggered by TE deficiency and impaired insulin sensitivity; moreover, LSG may accentuate TE deficiency. As such, a patient's Lcn2 and Zn-to-Cu ratio may be utilized as potential biomarkers of their TE status and metabolic improvement after LSG.

## 1. Introduction

Obesity is a chronic relapsing disorder resulting from excessive fat deposits that stimulate the release of inflammatory mediators such as tumour necrosis factor *α* (TNF-*α*) and interleukin 6 (IL-6), which predispose obese individuals to a proinflammatory state [1]; furthermore, obesity represents a substantial risk for type 2 diabetes, dyslipidaemia, ischemic heart disease, and other comorbidities [2]. While the low-grade inflammatory state caused by this disorder hinders the prevention and treatment of obesity and related complications, a laparoscopic sleeve gastrectomy (LSG) procedure has been shown to effectively achieve considerable weight loss and significantly improve obesity-related comorbidities [1, 3].

The article "Impact of Zinc to Copper Ratio and Lipocalin 2 in Obese Patients Undergoing Sleeve Gastrectomy" was published in 2022. Journal: Biomed Res Int.

Even though trace elements (TE) only account for 0.02% of total body weight, they are essential cofactors engaged in numerous metabolic pathways [4]. Specifically, zinc (Zn) and copper (Cu) act as structural ions in hormones, proteins, and receptors in various enzymatic reactions [5]; Zn has anti-inflammatory and antioxidant effects, and Cu is an integral component of many metalloenzymes such as ceruloplasmin and superoxide dismutase [4, 6]. Currently, there is insufficient research on the possible association between TE status and inflammation in obesity.

Lipocalin 2 (Lcn2), which is also known as neutrophil gelatinase-associated lipocalin (NGAL), is an adipokine belonging to the lipocalin family [7]. Lcn2 is a 25-KD *α*-glycoprotein that was originally identified in human neutrophils, which is abundantly secreted by adipocytes, renal cells, hepatocytes, and immune cells such as macrophages [7, 8]. Lcn2 overexpression in adipose tissue promotes the release of IL-6 inflammatory mediators and the NF-*κ*B ligand receptor activator, stimulates the conversion of preadipocytes into adipocytes, and impinges on nutrient metabolism and insulin resistance [9].

Accordingly, the primary aim of this study is to investigate the relationship between the TE status and specific inflammatory biomarkers—particularly serum Lcn2—in morbidly obese subjects before LSG and nine months after the procedure. Furthermore, a secondary aim of this study is to assess the Zn-to-Cu ratio value in patients with a detected TE deficiency.

## 2. Materials and Methods

This prospective study was conducted on 107 subjects with morbid obesity who were admitted to the surgery department at Alexandria University Hospital between January 2014 and August 2019. The selected participants were ≥20 years of age, with a body mass index (BMI) ≥ 40 kg/m^2^, fit for anaesthesia and surgery, plus committed to follow-up. Subjects suffering from gastroesophageal reflux disease, the presence of malignancy, and females using hormonal contraceptive pills were all excluded. A control group of 25 healthy volunteers with a BMI score lower than 25 and ranging in age from 28 to 45 years with a mean age of 37.5 ± 6.65 years was concurrently monitored.

The article "Impact of Zinc to Copper Ratio and Lipocalin 2 in Obese Patients Undergoing Sleeve Gastrectomy" was published in 2022. Journal: Biomed Res Int.

This study is registered at ClinicalTrials.gov ID (NCT04554082). All participants were subjected to a full clinical preoperative evaluation, in addition to an assessment of any associated comorbidities such as hypertension and diabetes mellitus. The research protocol was approved by the ethics committee (Protocol ID 0304707); and the ethical standards in the 1964 Declaration of Helsinki were observed. Informed written consent was obtained from all subjects included in this study.

### 2.1. Study Population

The subjects with morbid obesity were divided into three groups according to their respective body mass index (BMI): Group A had a BMI of 40–44.9 and included 47 subjects (i.e., 30 females and 17 males, mean BMI 42.92 ± 1.73 kg/m^2^, mean age 39.8 ± 10.8 years); Group B had a BMI of 45–49. 9 and included 31 subjects (i.e., 23 females and 8 males, mean BMI 47.32 ± 1.46 kg/m^2^, mean age 37.8 ± 9.7 years); Group C had a BMI that was ≥50 and included 29 subjects (i.e., 16 females and 13 males, mean BMI 51.8 ± 2.87 kg/m^2^, mean age 44.2 ± 11.84 years). The mean individual body weight reductions (Δ) were calculated for all three groups; and the differences between the subjects' baseline mean body weights and mean weights nine months postoperative were determined; then the mean Δ weight values of all groups were compared.

### 2.2. Laboratory Measurements

Fasting peripheral blood samples were collected from the participants prior to surgery and nine months postoperative. Each sample was divided into two tubes: EDTA for the complete blood count and the remainder in plastic tubes (W. Sarstedt, Inc., Princeton, NJ) to avoid trace-metal contamination. The serum samples were allowed to clot at room temperature for 30 minutes, then centrifuged at 4,000 × g.

Serum glucose, total cholesterol, HDL cholesterol, LDL cholesterol, triglycerides, total protein, albumin, serum CRP, serum iron (Fe), and ferritin were all measured using a Hitachi autoanalyzer 704 (Hoffman-La Roche Ltd., Basel, Switzerland); the serum samples were then stored at −80°C for further biochemical and TE analysis.

Serum insulin was measured using a solid-phase, chemiluminescence immunoassay (Immulite 2000; DPC, Siemens, NY). Insulin resistance (IR) was calculated using the Homeostasis Model Assessment (HOMA-IR) according to the following formula: fasting insulin (mU/L) × fasting glucose (mmol/L)/22.5.

Serum ceruloplasmin (Cp) levels were determined with a Beckman Array automated nephelometer. Zn and Cu levels were evaluated by an atomic absorption and emission spectrometer (Shimadzu 6401S, Shimadzu Biotech, Kyoto, Japan). The acetylene flow rate and burner height were both adjusted to achieve maximum absorbance signal with a slit of 0.5 nm, Zn at a 213.9 nm wavelength, and Cu at a 324.8 nm wavelength. The radiation sources were hollow cathode lamps (Shimadzu).

The article "Impact of Zinc to Copper Ratio and Lipocalin 2 in Obese Patients Undergoing Sleeve Gastrectomy" was published in 2022. Journal: Biomed Res Int.

The serum lipocalin-2 (Lcn2) was determined by ELISA with a DuoSet kit (DY1707 and DY1757, R&D Systems, Inc., Minneapolis, MN, USA). Serum leptin was analyzed by a Leptin ELISA Kit (MBS 700713) (Biosource, San Diego, CA, USA).

### 2.3. Surgical Technique

After establishing a capnoperitoneum, dissection began on the greater curvature approximately 5 cm from the pylorus. The greater curvature of the stomach was detached from the omentum and dissection extended until the left crus of the diaphragm was well-visualized, after which a 36 Fr gastric tube was advanced into the stomach. Beginning 5–6 cm lateral from the pylorus, a series of linear staples was applied toward the left of the lesser curvature vessels until reaching the gastric tube, then up to the angle of His. The resected stomach specimen was eradicated, and possible leakage was excluded by methylene blue testing [10].

### 2.4. Follow-Up Parameters

All studied subjects were followed-up within the first month for early postoperative complications such as bleeding or leakage. Concomitantly, the subjects' anthropometric measurements were assessed preoperative and three, six, and nine months postoperative; any preoperative comorbidities were appraised.

All participants received a regular course of postoperative medications, in addition to one A-to-Zinc multivitamin tablet, one 1,500 mg calcium tablet and one 10,000 IU vitamin D tablet every day. Compliance was emphasized through the use of a container with a known number of vitamin pills provided to the participants at the beginning of each month throughout the duration of the study, and the number of pills remaining from the previous month was counted; and compliance was assessed by comparing the total pills provided and those consumed by end of each month.

### 2.5. Data Analysis

All data were analyzed with the IBM® SPSS® version 20 software. The arithmetic mean and standard deviation were calculated for the categorized parameters using a chi-square test. A numerical data *t*-test was implemented to compare two groups, and an ANOVA test was utilised to compare more than two groups. A post hoc test using the Duncan method and small letters was employed to determine the level of significance between each group. The Spearman correlation coefficient was used to detect the correlation between different variables. Statistical correlations were calculated by Pearson's correlation test; *P* < 0.05 was considered significant.

The article "Impact of Zinc to Copper Ratio and Lipocalin 2 in Obese Patients Undergoing Sleeve Gastrectomy" was published in 2022. Journal: Biomed Res Int.

## 3. Results

All the morbidly obesity groups revealed a significantly decreased BMI at the end of the follow-up period, which was nine months postoperative; body weight reductions were most notable in Groups B and C, which were depicted by a baseline BMI ≥ 45. Moreover, most participants in the study groups achieved body weight reductions after bariatric surgery expressed as delta body weight change, as shown in Table 1. The analyzed metabolic variants and clinical characteristics of both the control group and the group with morbid obesity (including Groups A, B, and C) preoperative and at the end of the study period are delineated in Table 2.

The haematological parameters were within the laboratory normal ranges for a majority of the subjects, as shown in Table 3. Iron deficiency anaemia (IDA) was diagnosed by the presence of decreased haemoglobin (i.e., <13.5 g/dL in men and <12 g/dL in women), in addition to a mean corpuscular volume (MCV) below 80 fL, serum iron below 60 *μ*g/dL and ferritin below 30 ng/mL [11]. Because preoperative ferritin levels were elevated in all cases, they were not used to diagnose IDA; the diagnosis was therefore determined by evaluating haemoglobin, MCV, and serum iron levels. The mean preoperative MCV was 85.78 ± 5.9 fL, and the postoperative value was 84.67 ± 6.5 fL; furthermore, the preoperative mean corpuscular haemoglobin (MCH) was 30.1 ± 1.02 pg, and the postoperative estimate was 28.04 ± 1.7 pg.

Nine subjects (8.41%) in this study were found to have mild IDA preoperatively (i.e., two in Group A, three in Group B, and four in Group C), and five patients in Group C developed IDA postoperatively; consequently, a total of 14 (13.1%) subjects were found to have IDA postoperatively. A total of 11 (10.28%) subjects were diagnosed with serum-iron deficiency preoperatively (i.e., two in Group A, four in Group B, and five in Group C), and the prevalence increased to 17 (15.89%) postoperatively (i.e., five in Group A and eight in Group C); while preoperative serum iron levels ranged from 47.1–51.54 *μ*g/dL, these levels were reduced postoperatively and ranged from 38.3 to 49.87 *μ*g/dL. Consequently, a higher initial BMI and a significant loss of body weight led to a higher incidence of IDA, as shown in Figure 1.

Changes in Zn, Cu, and Cp serum concentration levels were observed preoperative and nine months postoperative, as shown in Table 4. Zn deficiency was defined as zinc levels < 70 *μ*g/dL for women and <74 *μ*g/dL for men; only 18 participants (16.82%) were diagnosed with Zn deficiency preoperative (i.e., six in Group A, four in Group B, and eight in Group C), and six participants developed de novo Zn deficiency (i.e., two in Group B and four in Group C), with an increased frequency to 24 (22.43%) postoperative. Cu deficiency was defined as copper levels < 70 *μ*g/dL; none of the subjects were diagnosed with Cu deficiency in the two consecutive measurements (i.e., pre- and postoperative). Similarly, there were no significant changes in the subjects' serum Cp levels throughout the study period.

The article "Impact of Zinc to Copper Ratio and Lipocalin 2 in Obese Patients Undergoing Sleeve Gastrectomy" was published in 2022. Journal: Biomed Res Int.

Delta body weight changes were correlated with clinical and laboratory parameters, such as TE and inflammatory biomarkers, and are shown in Table 5. Positive correlations between Lcn2 and Zn, the Zn-to-Cu ratio, and CRP were detected, as shown in Figure 2.

## 4. Discussion

Disturbances in the TE homeostasis of subjects with morbid obesity may be obscure due to the presence thereof in minute amounts and the lack of specific clinical features associated with certain TE deficiencies, which makes it difficult to differentiate between apparent and true TE deficits, particularly those of Zn and Cu [8, 12, 13]. The LSG is gaining popularity because it is a simple procedure with a negligible impact on most micronutrients—since it does not modify the absorption site thereof in the small intestine—and because it alleviates associated comorbidities to a greater extent than other bariatric procedures [14, 15].

IDA is identified by the presence of microcytosis and hypochromia (i.e., low MCV and MCH) and low serum iron and ferritin levels [11]. The results of the present study revealed a prevalence of preoperative serum-iron deficiency in 10.28% of the participants, which increased to 15.89% postoperatively; the 8.41% preoperative prevalence of IDA rose to 13. 1% after the LSG. Notably, serum iron levels were more reduced to a more significant degree in Group C than in Groups A and B in both the pre- and postoperative periods; this corresponds with the findings of Vargas-Ruiz et al., who reported an increased incidence of anaemia—from 10% to 26.6%—one year after a laparoscopic Roux-en-Y gastric bypass procedure [16].

Because ferritin is an inflammation-sensitive plasma protein (ISP), the significantly increased preoperative serum ferritin levels likely reflect the presence of subclinical inflammation [17, 18]; the study results also revealed significantly elevated preoperative levels of other ISPs such as CRP and serum Lcn2, compared to postoperative levels. It should be noted, however, that even though previous studies have reported a positive correlation between all ISPs including Cp and BMI, there was no significant difference in the Cp levels of the control and obese groups in the present study [19, 20]; this can be explained by an increased production of inflammatory cytokines and adipokines (i.e., leptin) in adipose tissue, which evoked hepatic ISP synthesis [20].

The article "Impact of Zinc to Copper Ratio and Lipocalin 2 in Obese Patients Undergoing Sleeve Gastrectomy" was published in 2022. Journal: Biomed Res Int.

Delta body weight change was 39.97 kg with the most significant drop in body weight of 49.35 kg observed in Group C. A negative association was observed between delta body weight change and Lcn2, CRP, leptin, and HOMA-IR, which implies that greater weight loss is accompanied by an ISP recession. Our results also revealed a correlation between Lcn2 and the CRP inflammatory biomarker, which is an established serum marker for chronic inflammation (*r* = 0.373, *P* = 0.012), as well as a correlation between both Δ body weight (*r* = −0.381, *P* = 0.0036) and HOMA-IR (*r* = 0.336, *P* = 0.01). This is in line with the assertion by Mosialou et al. that enhanced Lcn2 circulation associated with increased BMI in conjunction with development of insulin resistance is suggestive of metabolic dysregulation [21]; mounting evidence that inflammatory biomarkers either directly or indirectly influence obesity-related insulin resistance by impeding the stimulation of insulin-signalling receptors in pancreatic *β*-cells [22]; and the proposal by Rashad et al. that an obesity-related subclinical inflammatory state may elicit Lcn2 upregulation to counteract the effect of augmented adipose tissue inflammation and insulin resistance and may therefore serve a valuable role in energy metabolism [23].

Regarding Zn deficiency, only 16.82% of the study participants exhibited preoperative Zn deficiency, yet postoperative incidence increased to 22.43%. Preoperative Zn deficiency was more pronounced in participants from Groups B and C, which suggests an association between a higher BMI and a greater degree of Zn deficiency. Fukunaka et al. deduced that Zn deficiency in morbidly obese subjects is strongly correlated with oxidative stress, because Zn is involved in the synthesis of antioxidant enzymes and serves as a catalyst for various enzymes involved in lipid, carbohydrate, and protein metabolism [24, 25]. Another influential factor could be the intake of a poor-quality diet owing to the increased ingestion of processed foods that are low in micronutrients [26]. The observed increased postoperative incidence of Zn deficiency could be explained by standard multivitamin supplementation with insufficient zinc content [24]. This corresponds with the study by Sallé et al., which affirmed the existence of Zn deficiency in approximately 6.5% of obese subjects that increased to 18.8% one year after the LSG procedure and concluded that postoperative Zn malabsorption was attributed to bypassing the duodenum and proximal jejunum—the main sites for Zn absorption—and diminished the stomach yield of hydrochloric acid needed for Zn absorption and bioavailability [27, 28]. Gasteyger et al. also conducted a study on patients receiving standardized multivitamin preparation containing 5 mg of zinc and observed that Zn deficiency increased from 3% to 12% 6–24 months postsurgery [28].

The article "Impact of Zinc to Copper Ratio and Lipocalin 2 in Obese Patients Undergoing Sleeve Gastrectomy" was published in 2022. Journal: Biomed Res Int.

Zn supplementation is widely recognized as playing a role in reducing body weight, inflammatory markers, and insulin resistance in the treatment of obesity [25, 29]. In the present study, Zn was strongly correlated with both Lcn2 (*r* = 0.308, *P* = 0.01) and Δ body weight (*r* = 0.311, *P* = 0.011). Madan et al. stated that proinflammatory cytokines may stimulate the expression of genes encoding for zinc-transport proteins, such as Zip-14 and Zip-6, which promote the influx of Zn into cells and partially cause a false reduction in circulation [30]. Zn deficiency should therefore be strongly suspected in subjects with a low Zn-to-Cu ratio, particularly in those with insufficient Zn intake, or in cases of marginal deficiency in the absence of hypozincaemia [31].

Regarding the antagonistic effect of Zn and Cu, the absorption of each involves a competitive mechanism, and the surplus of one TE can therefore result in a deficiency of the other [29]. While the ideal serum Zn-to-Cu ratio is close to 1: 1, with Zn in balance with Cu in circulation, a small increase in Zn consumption in excess of the recommended amount may reduce Cu levels [25, 30]. The Zn-to-Cu ratio not only reflects the TE status of an individual but also plays a significant role in the pathogenesis of metabolic diseases. Our results revealed a positive correlation between the participants' delta body weight changes and Zn-to-Cu ratios (*r* = 0.46, *P* = 0.001).

It should be noted, however, that there was no significant difference between the subjects' pre- and postoperative serum Cu levels. This is contrary to the findings of Gletsu-Miller et al., who observed a Cu deficiency in approximately 10% of obese subjects 24 months after participating in bariatric surgery [32], and Kumar et al., who reported that postoperative Cu deficiency is rare [33]. Cu, which is principally stored in the liver, is released to maintain increased requirements of antioxidant enzymes and ceruloplasmin (Cp), a *α*-2 glycoprotein that incorporates more than 95% of the total Cu in circulation copper [34]; as a result, the level of circulating Cu is dependent on Cp and an ISP [35]. In this study, however, no significant difference was observed between the serum Cp levels in the control and morbid-obesity groups, and a Gelts close association was observed between the Zn-to-Cu ratio and Lcn2 (*r* = 0.371, *P* = 0.002); these results indicate that greater awareness of micronutrients concentrations—including those of multivitamins and TEs used in supplementation—is needed in postoperative plans after an LSG procedure has been performed.

The article "Impact of Zinc to Copper Ratio and Lipocalin 2 in Obese Patients Undergoing Sleeve Gastrectomy" was published in 2022. Journal: Biomed Res Int.

## 5. Conclusion

A relationship was observed between inflammatory biomarkers, such as Lcn2 and CRP, and TE levels in obese patients. Because metabolic conditions such as inflammatory status, stress, food intake, hormonal alterations, and anatomic variations following surgery may influence the labile Zn and Cu pools, the Zn-to-Cu ratio is more clinically superior than separately assessing TE concentration deficiencies. Furthermore, following a bariatric procedure, morbidly obese subjects will likely gain greater benefits by targeting systemic inflammation and important mineral and TE supplementation.

In this study, selected participants were morbidly obese with BMI ≥ 40 kg/m^2^ which may represent a limitation. Therefore, future studies will be needed on larger population of obese patients with variable range of BMI ≥ 30 kg/m^2^. Moreover, it is needed to study the relation of other TE and inflammatory biomarkers in obese patients undergoing bariatric surgery. Furthermore, prolonged follow-up periods are needed to monitor the long-term effects of bariatric procedures on TE status and to verify that sufficient TE supplements are prescribed to maintain appropriate TE levels. Also, additional prospective studies are needed to establish accurate TE supplementation, particularly of Zn, because no guidelines regarding optimal dosage currently exist.

## Figures and Tables

**Figure 1:** Percentage of trace element deficiency pre- and postoperative.

**Figure 2:** Correlation between serum Lcn2 and metabolic parameters.

**Table 1:** BMI and body weight changes in the control group and groups with morbid obesity (MO).

Group	No of subjects	Preoperative BMI (kg/m^2^)	Postoperative BMI (kg/m^2^)	Body weight preoperative	Body weight postoperative	Δ Body weight (kg)
Control	25	23.21 ± 1.45^a^	—	66.3 ± 14.37^a^	—	—
Group A	47	41.22 ± 1.73^b^	27.86 ± 2.67^a^	114.98 ± 11.74^b^	83.65 ± 8.94^a^	33.82^a^
Group B	31	47.32 ± 1.46^c^	34.31 ± 3.6^b^	131.34 ± 12.18^c^	88.39 ± 10.87^b^	36.79^b^
Group C	29	51.38 ± 2.87^c^	36.98 ± 3.87^b^	147.23 ± 14.68^d^	94.31 ± 10.54^c^	49.35^c^
ANOVA *P* value		36.5 0.001^∗^	9.85 0.003^∗^	29.8 0.001^∗^	6.12 0.013^∗^	5.85 0.022^∗^

Morbid obesity (MO) groups: Groups A, B, and C. ^∗^Statistically significant at *p* ≤ 0.05. Duncan's method was used to find the significant difference between two groups as follows: The same small letters indicate that there was no significant difference between the two groups, while the difference letters indicate that there was a significant difference between this two groups.

The article "Impact of Zinc to Copper Ratio and Lipocalin 2 in Obese Patients Undergoing Sleeve Gastrectomy" was published in 2022. Journal: Biomed Res Int.

**Table 2:** Clinical characteristics and metabolic variables in control group and group with morbid obesity (MO).

	Control group	MO group preoperative	MO group postoperative	ANOVA	*P* value
Systolic BP (mmHg)	130.5 ± 10^a^	146.0 ± 17.0^b^	132.0 ± 11.0^a^	8.03	0.002^∗^
Total cholesterol (mmol/L)	4.65 ± 0.35^a^	6.85 ± 0.41^b^	4.84 ± 0.33^a^	6.52	0.008^∗^
Triglycerides (mmol/L)	1.71 ± 0.47	2.10 ± 0.43	1.72 ± 0.34	2.15	0.158
HDL cholesterol (mmol/L)	1.41 ± 0.17^a^	1.20 ± 0.19^b^	1.35 ± 0.2^a^	4.25	0.011^∗^
LDL cholesterol (mmol/L)	2.68 ± 0.18^a^	3.73 ± 0.23^b^	2.81 ± 0.21^a^	4.01	0.026^∗^
HOMA-IR	1.31 ± 0.23^a^	2.64 ± 1.3^b^	1.44 ± 0.51^a^	6. 11	0.005^∗^
Leptin (ng/mL)	18.67 ± 6.78^a^	93.6 ± 11.9^b^	34.9 ± 16.7^c^	26.2	0.001^∗^
CRP (mg/L)	2.26 ± 0.76^a^	8.4 ± 5.91^b^	3.2 ± 2.98^c^	12. 3	0.007^∗^
Lipocalin 2 (*μ*g/L)	37.9 ± 16.8^a^	89.24 ± 13.8^b^	51.6 ± 19.73*c*	24.6	0.001^∗^
Albumin (g/dL)	4.41 ± 0.26	4.05 ± 0.21	3.95 ± 0.29	2.65	0.244

Subjects with morbid obesity (MO) group. ^∗^Statistically significant at *p* ≤ 0.05. Duncan's method was used to find the significant difference between two groups as follows: The same small letters indicate that there was no significant difference between the two groups, while the difference letters indicate that there was a significant difference between this two groups.

**Table 3:** Hemoglobin, iron, and ferritin in the control group and groups with morbid obesity (MO).

	Hb (gm/dL)		*P*1 value	Iron (*μ*g/dL)		*P*1 value	Ferritin (ng/mL)		*P*1 value
	Preoperative	Postoperative		Preoperative	Postoperative		Preoperative	Postoperative	
Control group	14.1 ± 1.32	—		97.82^a^ ± 14.7	—		89.65^a^ ± 21.47		
Group A	13.1 ± 1.01	12.43^a^ ± 1.1	0.107	81.75^b^ ± 29.81	89.67^a^ ± 31.42	0.107	112.67^b^ ± 40.39	87.25^a^ ± 30.7	0.011^∗^
Group B	12.8 ± 1.4	11.9^b^ ± 0.83	0.099	80.1^b^ ± 27.68	88.3^a^ ± 40.03	0.042^∗^	108.5^b^ ± 42.51	93.48^a^ ± 39.8	0.013^∗^
Group C	13.4 ± 2.5	11.56^b^ ± 1.89	0.046^∗^	67.73^c^ ± 23.55	75.54^b^ ± 39.84	0.013^∗^	157.56^c^ ± 68.5	105.78^b^ ± 34.18	0.002^∗^
ANOVA *P* value	3.01 0.113	5.21 0.031^∗^		21.65 0.001^∗^	5.21 0.013^∗^		15.6 0.001^∗^	10.5 0.008^∗^	

Morbid obesity (MO) groups: Groups A, B, and C. P1 comparison between pre and postoperative. ANOVA to compare between the different groups at the same time. Duncan's method was used to find the significant difference between two groups as follows: The same small letters indicate that there was no significant difference between the two groups, while the difference letters indicate that there was a significant difference between this two groups.

**(a):** 

	Cu (*μ*g/dL)		*P*1 value	Zn (*μ*g/dL)		*P*1 value
	Preoperative	Postoperative		Preoperative	Postoperative	
Control group	142.34 ± 19.56^a^	—		128.67 ± 16.56^a^	—	
Group A	130.9 ± 32.82^a^	122.2 ± 31.36^a^	0.085	101.01 ± 28.08^b^	78.57 ± 24.06^a^	0.003^∗^
Group B	119.63 ± 29.57^b^	113.67 ± 29.45^b^	0.066	87.98 ± 22.17^c^	82.34 ± 20.67^b^	0.104
Group C	113.78 ± 21.97^b^	110.75 ± 29.81^b^	0.145	81.88 ± 20.01^c^	9	0.098
ANOVA *P* value	21.3 0.001^∗^	5.21 0.031^∗^		26.5 0.001^∗^	5.04 0.039^∗^	

**(b):** 

	Zn-to-Cu ratio		*P*1 value	Ceruloplasmin (mg/dL)		*P*1 value
	Preoperative	Postoperative		Preoperative	Postoperative	
Control group	0.9 ± 0.05^a^	—		30.58 ± 8.89	—	
Group A	0.78 ± 0.05^b^	0.64 ± 0.09	0.041^∗^	31.23 ± 12.78	28.77 ± 10.9	0.069
Group B	0.74 ± 0.01^b^	0.72 ± 0.02	0.526	28.73 ± 9.55	26.87 ± 8.76	0.104
Group C	0.72 ± 0.02^b^	0.63 ± 0.04	0.023^∗^	28.23 ± 10.78	25.68 ± 9.44	0. 21
ANOVA *P* value	6.01 0.029^∗^	2.85 0.141		2.07 0.331	1.68 0.411	

Morbid obesity (MO) groups: Groups A, B, and C.

The article "Impact of Zinc to Copper Ratio and Lipocalin 2 in Obese Patients Undergoing Sleeve Gastrectomy" was published in 2022. Journal: Biomed Res Int.

**Table 5:** Correlation between delta change in body weight and other laboratory findings.

Δ Body weight (kg)^#^	Correlation coefficient “*r*”	*P* value
Lcn2	-0.381	0.0036^∗^
CRP	-0.373	0.012^∗^
Systolic blood pressure	0.107	0.113
Zn-to-Cu ratio	0.46	0.001^∗^
Zn	0.311	0.011^∗^
Cu	0.19	0.236
Ferritin	0.201	0.107
Iron	0.156	0.136
HOMA-IR	-0.355	0.013^∗^
Leptin	-0.298	0.014^∗^

## Data Availability

The data will be available upon request.

## Abbreviations

BMI: Body mass index
Cp: Ceruloplasmin
CRP: C-reactive protein
Cu: Copper
Fe: Iron
IR: Insulin resistance
ISP: Inflammation-sensitive plasma protein
Lcn2: Lipocalin 2
LSG: Laparoscopic sleeve gastrectomy
TE: Trace elements
Zn-to-Cu ratio: Zinc-to-copper ratio.

## Additional Points

*Key Points*. Obesity is characterized by excess accumulation of macronutrients in the adipose tissues which promotes the release inflammatory mediators and predisposes to proinflammatory state and oxidative stress. Therefore, assessment of trace element status in obesity should be done in conjunction with inflammatory response. Evaluation of zinc-to-copper ratio is more efficient in measurement of trace elements status than either element alone in obesity. Lipocalin 2, besides its role as an inflammatory biomarker, is also involved in regulation of body metabolism and may be in micronutrient metabolism.
